# Optimizing laser cladding powder injection parameters to shape bioactive glass nano-coated zirconium oxide for biomedical application

This article has been retracted.

**DOI:** 10.1016/j.heliyon.2024.e25277

**Published:** 2024-01-26

**Authors:** Sathish T, Jayant Giri, R. Saravanan

**Affiliations:** a Department of Mechanical Engineering, Saveetha School of Engineering, Saveetha Institute of Medical and Technical Sciences (SIMATS), Saveetha University, Chennai, Tamil Nadu, India; b Department of Mechanical Engineering, Yeshwantrao Chavan College of Engineering, Nagpur, Maharashtra, India

**Keywords:** Biomaterials, Biomedical, Laser power, Taguchi method, Compressive strength, Microhardness, Wear

## Abstract

Human body is highly sensitive and repairing often incurs pain and expenses. Strength of the materials degraded by poor joint (either weld or link). New material technology is proposed many biomaterials for repairing bone and tissue and also many bio-implantation applications. Especially bioactive material like bioactive glass is used for biomedical applications for replacement and repairing organs in human body. This research work focuses on suggesting material of S53P4 bioactive glass Nano-coated Zirconium dioxide for manufacturing artificial knee implant for fixing in human body. The substrate of Zirconium dioxide is Nano-coated with S53P4 bioactive glass by means of laser cladding process. The laser cladding process parameters were optimized by Taguchi method to enhance mechanical properties like compressive strength, wear resistance and microhardness of Zirconium dioxide implant material. The key parameters like Laser Power (1 kW, 2 kW, 3 kW and 4 kW), beam diameter (2 mm, 3 mm, 4 mm and 5 mm), powder feed rate (10 g/min, 15 g/min, 20 g/min and 25 g/min) and scanning speed (3 mm/s, 4 mm/s, 5 mm/s and 6 mm/s) were considered. The optimal parameters result the higher compressive strength and microhardness are obtained as 373 MPa and 898.37 HV0.2 and minimum wear volume is attained as 0.148 mm^3^ in the Nano-coated implant material.

## 1 Introduction

In past years the replacement of human bone, solving of spinal problems, distressing injuries, joint problems and tissue-related problems are complicated to rectify. Recently a lot of biomaterials is involved to give the solution of the human normal life [1]. Biomaterials are focused on making prostheses and implants for medical applications such as the recovery of the original structure of the human body. Biomaterials are influenced by the fabrication of spinal parts, stent making, concentration in tissue generation and dental application [[2], [3], [4]]. Sometimes biomaterials are used in the total replacement of hip and knee joints. Biomaterials need a vast study for their properties such as mechanical, biological, biocompatibility and thermal properties [5]. Generally, the expectations focused on biomaterials are to meet the requirements while the parts are placed in the human body. The biomaterials possess very good properties and are non-toxic, biocompatible, non-carcinogenic and non-allergenic conditions [[6], [7], [8]]. Biomaterials are to be classified based on their function, there are classified into three generations such as old generation, mid-generation and the new generation. In the old generation, the biomaterials meet the requirements of replaced tissue based on mechanical and biological properties [[9], [10], [11]]. These old generation biomaterials are not affected by influencing biological and chemical changes while in function in the human body. The biological environment does not affect the action and reaction of mid-generation biomaterials, these materials are used to encourage new bone generation with controllable function [[12], [13], [14]]. New generation biomaterials are very good properties, devices made on these materials are degraded constantly and surrogated by a livelihood multitude of tissues [15].

Due to their excellent properties to meet the requirements of medical applications of biomaterials include glasses, ceramics, metals and polymers [16]. Compared to all materials polymers are a flexible group of biomaterials, it can satisfy industrial applications namely food production units, farming, pharmaceutical applications and biomedical sectors [[17], [18], [19]]. Generally, the polymers are grouped into two categories namely synthetic polymer and natural polymer. Natural polymers are used to combine one another, it is formed new materials and improve the properties and ease of workability [[20], [21], [22]]. Normally the natural polymers with ceramics fillers combo offered better mechanical properties. Ceramics fillers typically known as bioactive glasses (BGs), it is used in medical applications [23]. Bioactive glass is extremely used in tissue engineering and bone replacement in the human body, a combination of titanium, zirconium, magnesium and stainless steel with bioactive glass offered better mechanical properties for the implants [[24], [25], [26]]. These combinations are used to replacement of joints, spinal, dental applications etc. Particularly Zirconium dioxide with bioactive glass combination is used to total replacement of knee in the human body [27]. In recent years bioactive glass is generated in different categories of applications, BGs containing the counteractive ions namely strontium and magnesium [28]. Based on the sodium or borate-containing bioactive glass must be favourable for bioactivity and biological response. Recently bioactive glass possesses antibacterial properties when the combination of Cu, Zn, and Ag ions was included in BGs [29]. Laser technology has recently been used vastly for surface alteration of various materials, to its high-performance beam delivery, extreme energy occurred and high consistency. Laser cladding is a manufacturing technique that utilises a laser beam to apply a metallic substance onto a surface, serving as the primary heat source. The substance undergoes a process of melting and fusion with the surface, resulting in increased hardness and wear resistance compared to the base material. Material involving in the laser cladding is S53P4 Bioactive Glass Nanocoated Zirconium oxide (ZrO_2_), that is a substance and compatible with living organisms. Laser operations on the surface of the materials are known as Laser surface remelting or laser cladding; this operation highly improves the surface of the materials [30,31]. The laser cladding process is widely used to make surface modifications with different kinds of coatings, the laser cladding process offered extreme production competence and deposition can be easy to controllable. Inert argon gas is used in the laser cladding process to protect the oxidation and carry coating powder to the substrate at the time of laser beam directly to the metal surface [32]. Laser welding highly biocompatible and applied widely in working with biomedical devices and implant materials and most of the studies delt with mechanical strengths of the joints [33]. [34] used laser cladding for coating bioinert TiC ceramic on Ti6Al4V substrate, causes three times higher wear resistance than uncoated one [35]. studied the influence of various process parameters of Laser surface remelting process for Ti alloys [36]. validated the possibility of laser cladding to create bioactive glass coatings on alumina/zirconia ceramic acetabular cups used in hip joint prostheses. The hybrid powers of CeO_2_, TiC and ZrO2 on Ti6Al4V and observed the wear and micro-hardness. The influence of CeO_2_ powers was investigated [37]. [[38], [39], [40]] experimentally found that micro-hardness and wear resistance of samples influenced by the material used for cladding and recommended the optimization to maximize the microhardness and minimize the wear in the cladded joints [41]. utilized Taguchi orthogonal experimental design for optimizing the laser cladding processing parameters [42]. highlighted in his review that many researchers focused their studies on laser cladded titanium alloys and their potential applications. The gap analysis reveals that laser cladding with S53P4 Bioactive Glass Nanocoated Zirconium oxide in bio implant application and optimizing process parameters for compressive strength, wear and micro hardness not reported in the literature so far and this study is unique and novel. As most of the issues of implant failures at joints due to compressive load, poor surface hardness and lack of wear resistance at joints [43]. That is most important properties for knee bone implants are compressive strength, surface hardness and wear [44]. So, the present work aims to suggest the material of S53P4 Bioactive Glass coating on zirconium dioxide material with the aid of a laser cladding process by optimizing most responsible process parameters with the help of the Taguchi optimization technique to produce knee implant. The objective of this research to enhance the quality of Laser cladding of Nanocoating of S53P4 Bioactive Glass on Zirconium oxide substrates by optimizing the process parameters such as Laser Power, Beam diameter, Powder Feed rate and Scanning Speed to shape to achieve the key properties of knee bone implant.

### 1.1 Experimental procedure

This work considered S53P4 Bioactive Glass as a coating material, it possesses 99.2 % purity, 1.5 g/cm^3^ density and 50 μm of particle size. S53P4 Bioactive Glass is a mixture of high purity CaO:SiO_2_:P_2_O_5_ formation. This bioactive glass was purchased from Nano Research Elements, Haryana with the required quantity. Making knee implant using zirconium dioxide as the substrate of this investigation, the zirconium dioxide is procured from Horizon metal and alloys, Mumbai with the required quantity. Zirconium dioxide plate 6 mm thickness and 50 × 50 mm^2^ of size substrate is used for this investigation. The substrates need no special surface finishing after standard machining.

Coating of the S53P4 Bioactive Glass on zirconium dioxide substrate is carried out by using of laser cladding powder injection process. In the laser cladding technique, the bioactive glass powder particles are blown with a carrier gas through a powder injection nozzle over the zirconium substrate. This process is conducted under the laser beam action as shown in Fig. 1. Rigid and stationary high-power laser energy is directed to the top surface of the substrate. Striking of the laser beam is used to melt the bioactive glass particles and formed a molten pool on the substrate surface. At that time the shielding inert gas is passed on the substrate for avoiding oxidation in the interaction zone. In this experimental Nd: YAG laser source is used with k = 1064 nm wavelength. Using expanding and collimating optics with 400 lm core diameter optical fibre arrangements. Excellent focal of the laser beam is achieved through using of a lens with 90 mm focal length, different diameters of beam spot such as 2 mm, 3 mm, 4 mm and 5 mm are used. Inert argon gas support conveys and injects the powder particles of the bioactive glass into the interaction zone. A 402 TS micro-hardness tester (HDNS, Shanghai, China) applied 0.2 g of force for 30 s to test the micro-hardness. The wear volume indicator was used to interpret the wear resistance. A UMT-2 high load scratch tester (Bruker, Billerica, MA, USA) was used to measure the wear volume by continuously applying reciprocating scratch for 30 min. Next, using white light interferometry, the 3D morphology of each sample's scratch surface was determined. Each sample's wear volume was then measured [39,41]. The computes assisted universal testing machine of model INSTRON E−3000 was utilized to characterizes the samples for compressive strength.

**Fig. 1:** Experimental setup for laser cladding powder injection process.

The substrate was placed under the laser head and using different parameters the laser cladding coating was carried out in different zirconium dioxide plates. Different parameters are used such as laser power 1 kW, 2 kW, 3 kW, and 4 kW, beam diameter 2 mm, 3 mm, 4 mm and 5 mm, Powder feed rate 10 g/min, 15 g/min, 20 g/min and 25 g/min and scanning speed 3 mm/s, 4 mm/s, 5 mm/s and 6 mm/s. After coating the compressive strength, microhardness and wear tests are conducted on the substrate plates. Table 1 presented the Process parameters and their levels of the laser cladding process.

**Table 1:** Different Process parameters and their levels of the laser cladding process.

S. No	Parameters	Level 1	Level 2	Level 3	Levels 4
1.	Laser Power (kW)	1	2	3	4
2.	Beam diameter (mm)	2	3	4	5
3.	Powder Feed rate (g/min)	10	15	20	25
4.	Scanning Speed (mm/s)	3	4	5	6

## 2 Results and discussions

Using of laser cladding process, the mechanical properties of the S53P4 Bioactive glass-Nano-coated ZrO_2_ was highly enhanced. Extreme compressive strength and microhardness of the fabricated biomaterial knee implant were found as 373 MPa and 898.37 HV0.2. Similarly, the minimum wear volume was obtained as 0.148 mm^3^. Higher laser power, powder feed rate and moderate beam diameter and scanning speed offered good mechanical properties; it was presented in Table 2.

**Table 2:** Experimental summary of Laser cladding process and output.

Exp. No	Laser Power (kW)	Beam diameter (mm)	Powder Feed rate (g/min)	Scanning Speed (mm/s)	Compressive strength (MPa)	Microhardness (HV0.2)	Wear volume (mm^3^)
1	1	2	10	3	256	740.61	0.217
2	1	3	15	4	212	695.74	0.187
3	1	4	20	5	287	780.34	0.244
4	1	5	25	6	315	835.49	0.321
5	2	2	15	5	186	665.87	0.169
6	2	3	10	6	169	610.18	0.148
7	2	4	25	3	358	894.32	0.421
8	2	5	20	4	340	870.81	0.398
9	3	2	20	6	221	709.24	0.198
10	3	3	25	5	364	895.72	0.427
11	3	4	10	4	269	765.39	0.217
12	3	5	15	3	365	800.89	0.416
13	4	2	25	4	373	898.37	0.451
14	4	3	20	3	356	881.64	0.383
15	4	4	15	6	289	783.28	0.254
16	4	5	10	5	361	889.83	0.311

### 2.1 Compressive strength analysis

Employing DOE analysis, a larger is better condition was selected for analyzing of precedence of parameters in compressive strength analysis as presented in Table 3. Among four parameters involved in the laser cladding process, the powder feed rate parameter was highly influenced go behind laser power, beam diameter and scanning speed parameters. All the priority level parameters were concluded based on rank order and delta value obtained in the DOE analysis. In the compressive strength analysis, the optimal parameters were obtained as follows: 4 kW of laser power, 5 mm of beam diameter 25 g/min of powder feed rate and 3 mm/s of scanning speed.

**Table 3:** Response Table for Signal to Noise Ratios (Compressive strength analysis).

Level	Laser Power (kW)	Beam diameter (mm)	Powder Feed rate (g/min)	Scanning Speed (mm/s)
1	48.45	47.97	48.12	50.38
2	47.91	48.33	48.10	49.30
3	49.49	49.51	49.43	49.23
4	50.71	50.75	50.93	47.66
Delta	2.79	2.78	2.83	2.72
Rank	2	3	1	4

Increasing laser power from 1 kW to 4 kW highly enhanced the compressive strength of the knee implant as shown in Fig. 2, which indicates higher laser power extremely melt the bioactive glass powder and obtained excellent Nano-coating on the ZrO_2_ substrate. Similarly, the larger diameter of the beam induced a high rate of deposition of bioactive glass into the implant material and it improved the mechanical properties. The beam diameter of 5 mm offered higher compressive strength compared to other sizes of bream diameter. The elevated powder feed rate offered good compressive strength, increasing of powder feed rate from 10 g/min to 25 g/min boost the compressive strength appreciably. Compared to these three parameters, the lower level of scanning speed parameter recorded high compressive strength, if increasing the scanning speed, the compressive strength was reduced constantly. The delta value is high the ranking will be high. The data value implied the contribution of the parameters in modifying the compressive strength. From this table it can be understood the factor and at which level is suitable for maximize the compressive strength to perform cladding. In this case Powder Feed rate is Rank as its delta value is 2.83, in which level 4 has higher signal to noise ratio as 50.93 than other levels. So, Powder Feed rate at level 4 is optimal, similarly, Laser Power is rank 2 (delta = 2.79) and level 4 S/N ratio is 50.71 and so on.

**Fig. 2:** Main effects plots for S/N ratios for Compressive strength analysis.

A higher F value denoted the higher contribution percentage of the parameter in compressive strength analysis; it was presented in Table 4. From the ANOVA analysis, the powder feed rate was extremely contributed such as 25.49 % followed by beam diameter of 22.25 %, laser power of 20.56 % and scanning speed of 17.87 %.

**Table 4:** Analysis of Variance for Compressive strength analysis.

Source	DF	Seq SS	Contribution	Adj SS	Adj MS	F-Value	P-Value
Regression	4	62586	86.16 %	62586	15646.5	17.13	0.000
Laser Power (kW)	1	14933	20.56 %	14933	14933.1	16.35	0.002
Beam diameter (mm)	1	16160	22.25 %	16160	16159.6	17.69	0.001
Powder Feed rate (g/min)	1	18514	25.49 %	18514	18513.6	20.27	0.001
Scanning Speed (mm/s)	1	12980	17.87 %	12980	12979.5	14.21	0.003
Error	11	10049	13.84 %	10049	913.6		
Total	15	72635	100.00 %				

Regression Equation

(1) Compressive strength (MPa) = 135.4 + 27.32 Laser Power (kW) + 28.43 Beam diameter (mm) + 6.08 Powder Feed rate (g/min) - 25.48 Scanning Speed (mm/s)

The prediction model for compressive strength is furnished in equation (1). This can be utilized to predict the values for the unexperimented combinations of parameters. In compressive strength analysis, all parameters were statistically significant; it is illustrated in Fig. 3. Pareto chart visibly presents the parameters influence in compressive strength analysis; powder fed rate was 90 % statistically significant. Beam diameter was 85 % statistically significant, the laser power was 80 % statistically significant and scanning speed was 76 % statistically significant.

**Fig. 3:** Pareto chart of standardized effects (Compressive strength analysis).

Fig. 4 illustrates the compressive strength analysis with two parameters involved. Maximum laser power of 4 kW and 2 mm of beam diameter was registered high compressive strength as shown in Fig. 4 (a). Higher powder rate (25 g/min) and minimum beam diameter (2 mm) recorded excellent compressive strength as illustrated in Fig. 4 (b). Similarly, maximum powder rate (25 g/min) and moderate scanning speed (4 mm/s) offered good compressive strength as shown in Fig. 4 (c). Fig. 4 (d) depicts that Moderate scanning speed (4 mm/s) and maxim higher laser power (4 kW) provided exceptional compressive strength.

**Fig. 4:** Parallel pot for compressive strength analysis: (a) Laser power vs. Beam diameter (b) Beam diameter vs. Powder feed rate (c) Powder feed rate vs. Scanning speed (d) Scanning speed vs. laser power.

### 2.2 Microhardness analysis

The main aim was to maximize the microhardness of the knee implant, hence considered the larger is a better state in DOE analysis. All the parameter values of the laser cladding process were transformed into an S/N ratio, which was presented in Table 5. Based on the rank order and delta values were illustrated the priority of the process parameters in the microhardness analysis. Powder feed rate was the highly influenced parameter followed by laser power, scanning speed and beam diameter. Optimal parameters obtained in the microhardness analysis as laser power of 4 kW, a beam diameter of 5 mm, powder feed rate of 25 g/min and scanning speed of 3 mm/s.

**Table 5:** Response Table for Signal to Noise Ratios (Microhardness analysis).

Level	Laser Power (kW)	Beam diameter (mm)	Powder Feed rate (g/min)	Scanning Speed (mm/s)
1	57.63	57.49	57.44	58.35
2	57.50	57.63	57.32	58.10
3	57.95	58.11	58.14	58.09
4	58.71	58.57	58.90	57.26
Delta	1.21	1.09	1.58	1.09
Rank	2	4	1	3

Increasing laser power from 1 kW to 4 kW improves the microhardness of the knee implant. Higher laser power (4 kW) offered maximum microhardness values as shown in Fig. 5. A similar trend was observed in the beam diameter influences such as increasing of beam diameter from 2 mm to 5 mm recorded maximum microhardness values. A higher powder feed rate of 25 g/min provided excellent microhardness values. Increasing scanning speed decreases the microhardness values, the minimum value (3 mm/s) of scanning speed enhances the microhardness. There will be a high ranking if the delta value is high. The data value suggested how the parameters affected the compressive strength. This table makes it clear which factor to use and at what level to apply cladding in order to maximize compressive strength. As the delta value in this instance is 1.58, the Powder Feed rate is Rank, and level 4 has a greater signal-to-noise ratio than the other levels at 58.90. Therefore, the level 4 powder feed rate is optimum. In a similar vein, the level 4 S/N ratio is 58.71, the laser power is rank 2 (delta = 1.21), and so on.

**Fig. 5:** Main effects plots for S/N ratios for Microhardness analysis.

A higher contribution (33.73 %) was induced by powder feed rate in the microhardness analysis, it was presented evidently in Table 6. The other three parameters were contributed as follows laser power 17.51 %, beam diameter 16.37 % and scanning speed 12.73 %. The P-value of all parameters were observed less than 0.05 it was satisfied the selected parameters were statistically significant.

**Table 6:** Analysis of Variance for Microhardness analysis.

Source	DF	Seq SS	Contribution	Adj SS	Adj MS	F-Value	P-Value
Regression	4	101890	80.33 %	101890	25472	11.23	0.001
Laser Power (kW)	1	22207	17.51 %	22207	22207	9.79	0.010
Beam diameter (mm)	1	20764	16.37 %	20764	20764	9.15	0.012
Powder Feed rate (g/min)	1	42778	33.73 %	42778	42778	18.86	0.001
Scanning Speed (mm/s)	1	16141	12.73 %	16141	16141	7.12	0.022
Error	11	24952	19.67 %	24952	2268		
Total	15	126842	100.00 %				

Regression Equation

(2) Microhardness (HV0.2) = 564.8 + 33.3 Laser Power (kW) + 32.2 Beam diameter (mm) + 9.25 Powder Feed rate (g/min) - 28.4 Scanning Speed (mm/s)

The prediction model for Microhardness at the joint is furnished in equation (2). This can be utilized to predict the values for the unexperimented combinations of parameters. Fig. 6 illustrates the minimum to the maximum influence of parameters in microhardness analysis through Pareto chart analysis. This analysis proves that all the parameters were statistically significant predictor C was extremely influenced in the microhardness analysis. Selected parameters crossed the mean line that specifies all parameters were statistically significant.

**Fig. 6:** Pareto chart of standardized effects (Microhardness analysis).

Fig. 7 exemplifies the relationship between the two parameters for the response of microhardness in this analysis. A higher microhardness value was observed by the correlation of 2 kW laser power and 2 mm of beam diameter as shown in Fig. 7 (a). The powder feed rate of 25 g/min and 2 mm of beam diameter was highly influenced to maximize the microhardness value as shown in Fig. 7 (b). Scanning of 3 mm/s and 25 g/min of powder feed rate offered a high microhardness value as shown in Fig. 7 (c). Maximum laser power 4 kW and 5 mm/s scanning speed combination offered maximum microhardness value, it was presented in Fig. 7 (d).

**Fig. 7:** Trajectory pot for microhardness analysis: (a) Laser power vs. Beam diameter (b) Beam diameter vs. Powder feed rate (c) Powder feed rate vs. Scanning speed (d) Scanning speed vs. laser power.

### 2.3 Wear volume analysis

Wear volume analysis and the parameters influence were presented in Table 7, powder feed rate was highly influenced it was observed through rank order and delta value. The second priority parameter was observed as scanning speed, third priority parameter as beam diameter and fourth priority parameter as laser power. Optimal parameters were concluded as 1 kW of laser power, 2 mm of beam diameter, 10 g/min powder feed rate and 6 mm/s scanning speed.

**Table 7:** Response Table for Signal to Noise Ratios (Wear volume analysis).

Level	Laser Power (kW)	Beam diameter (mm)	Powder Feed rate (g/min)	Scanning Speed (mm/s)
1	12.489	12.424	13.320	9.185
2	11.888	11.721	12.382	10.688
3	10.587	11.235	10.664	11.308
4	9.325	8.909	7.923	13.109
Delta	3.164	3.515	5.397	3.924
Rank	4	3	1	2

Increasing laser power, beam diameter and powder feed rate levels increases the wear volume as shown in Fig. 8. Minimum levels extremely reduced the wear volume, contrarily higher scanning speed offered minimum wear volume. A high delta value corresponds to a high ranking. How the parameters influenced the compressive strength was indicated by the data value. If you want to maximize compressive strength, this table will show you which factor to utilise and at what level to apply cladding. In this case, level 1 has a higher signal-to-noise ratio (12.489) than the other levels because to the delta value of 5.397, the Powder Feed rate being Rank 1. The next rank is for Scanning Speed (rank 2) as delta = 1.21, laser power, level 4 S/N ratio is 13.109. like the way other ranks too.

**Fig. 8:** Main effects plots for S/N ratios for Wear volume analysis.

Results of wear volume analysis is illustrated in Table 8, in which the powder feed rate was extremely influenced it was contributed as 42.46 %. Scanning speed contribution was observed as 20.44 %, laser power contribution was recorded as 14.97 % and beam diameter contribution was 11.25 %. In wear volume analysis, P- values of all parameters were registered as less than 0.05; hence this investigation was statistically significant.

**Table 8:** Analysis of Variance for Wear volume analysis.

Source	DF	Seq SS	Contribution	Adj SS	Adj MS	F-Value	P-Value
Regression	4	0.14837	89.13 %	0.14837	0.037092	22.55	0.000
Laser Power (kW)	1	0.02492	14.97 %	0.02492	0.024922	15.15	0.003
Beam diameter (mm)	1	0.01873	11.25 %	0.01873	0.018727	11.39	0.006
Powder Feed rate (g/min)	1	0.07069	42.46 %	0.07069	0.070686	42.97	0.000
Scanning Speed (mm/s)	1	0.03403	20.44 %	0.03403	0.034031	20.69	0.001
Error	11	0.01809	10.87 %	0.01809	0.001645		
Total	15	0.16646	100.00 %				

Regression Equation

(3) Wear by volume (mm^3^) = 0.0798 + 0.03530 Laser Power (kW) + 0.03060 Beam diameter (mm) + 0.01189 Powder Feed rate (g/min) - 0.04125 Scanning Speed (mm/s)

The prediction model for Microhardness at the joint is furnished in equation (3). This can be utilized to predict the values for the unexperimented combinations of parameters. The Pareto chart simply demonstrates the influence of parameters and preference as shown in Fig. 9. In this analysis, predictor C such as powder feed rate was highly influenced followed by scanning speed, laser power and beam diameter. Among all parameters, beam diameter was a low contribution, but it was statistically significant.

**Fig. 9:** Pareto chart of standardized effects (Wear volume analysis).

Minimum wear volume was obtained with the effect of correlation of two parameters as shown in Fig. 10. Laser power of 2 kW and 3 mm of beam diameter correlation reduce the wear volume as shown in Fig. 10 (a). Minimum powder feed rate (10 g/min) and 3 mm beam diameter offered minimum wear volume; it was illustrated in Fig. 10 (b). Higher scanning speed (6 mm/s) and minimum powder feed rate (10 g/min) recorded minimum wear volume as shown in Fig. 10 (c). a lower level of laser power 2 kW and maximum scanning speed of 6 mm/s provided minimum wear volume of the implant as shown in Fig. 10 (d).

**Fig. 10:** Heat map pot for wear volume analysis: (a) Laser power vs. Beam diameter (b) Beam diameter vs. Powder feed rate (c) Powder feed rate vs. Scanning speed (d) Scanning speed vs. laser power.

The diagrams visible in Fig. 3, Fig. 4, Fig. 6, Fig. 7, Fig. 9 to show the percentage of contribution of parameters towards the research objective. These data can be utilized to personalize the results by rapid and/or fine tuning of these parameters. The high contributed parameters are more sensitive one can use them for rapid changes vice versa.

The knee bone implants properties requirements were widely investigated with various materials and methods. The compressive strength of UHMWPE and carbon reinforced polyethylene tibial based knee implants exhibited good stability at 150 and 300 MPa respectively [45]. The compressive strength requirement for Knee implant was considered as 220 MPa by considering 80 kg average body weight, gait [46,47]. In this investigation the optimal compressive strength as 373 MPa was recorded [48]. reported that micro hardness of knee bone implant material of Lithography-based ceramic recorded as 559 ± 27 HV. The proposed laser cladded sample specimen for knee bone achieved 898.37 HV [49]. reported that the alternate material of Cobalt–chromium–molybdenum alloy for knee bone implant recorded the wear volume as 0.79 mm. but in this investigation the minimum wear volume attained was 0.148 mm^3^. Hence the aim of optimizing laser cladding process parameters for nano coating of S53P4 bioactive glass on the substrate of Zirconium dioxide for suggesting alternate material for knee implant was achieved.

## 3 Conclusion

The optimization of by laser cladding process parameters such as Laser Power, Beam diameter, Powder Feed rate and Scanning Speed to shape the Zirconium dioxide-Nano-coated S53P4 bioactive glass for knee implant applications was discussed. The experiments were made at16 different setting as per Taguchi L16 orthogonal array. The samples were characterized in terms of Compressive strength, Microhardness and Wear. The followings are findings.

• The samples which laser cladded at 4 kW of laser power, 5 mm of beam diameter 25 g/min of powder feed rate and 3 mm/s of scanning speed recorded maximum compressive strength of 373 MPa and microhardness of microhardness 898.37 HV0.2. the power feed rate factor influencing higher than other factors may be considered for rapid tuning of process. The scanning speed is recorded lower contributions but significant (As p < 0.05), so this parameter could be used for fine tuning of process.
• In case of compressive strength Compressive strength has to be modified by different parameters contribution such as powder feed rate of 25.49 % followed by beam diameter of 22.25 %, laser power of 20.56 % and scanning speed of 17.87 %. For the micro hardness a higher contribution (33.73 %) was observed by powder feed rate followed by laser power 17.51 %, beam diameter 16.37 % and scanning speed 12.73 %.
• In wear volume analysis, optimized parameters were obtained as 1 kW of laser power, 2 mm of beam diameter; 10 g/min powder feed rate and 6 mm/s scanning speed. The contribution of each parameter in the wear volume analysis was registered as 42.46 % of powder feed rate 20.44 % of scanning speed, 14.97 % of laser power and 11.25 % of the beam diameter.

## CRediT authorship contribution statement

**Sathish T:** Writing – original draft, Visualization, Validation, Supervision, Methodology, Investigation, Data curation, Conceptualization. **Jayant Giri:** Writing – review & editing, Supervision, Software, Data curation, Conceptualization. **R. Saravanan:** Writing – review & editing, Validation, Resources, Project administration, Methodology, Investigation, Formal analysis.

## Declaration of competing interest

The authors declare that they have no known competing financial interests or personal relationships that could have appeared to influence the work reported in this paper.

## References

[1] Faria D., Henriques B., Souza A.C., Silva F.S., Carvalho O. (2020). Laser-assisted production of HAp-coated zirconia structured surfaces for biomedical applications. J. Mech. Behav. Biomed. Mater..

[2] Jaiswal Satish, Dubey Anshu, Lahiri Debrupa (2020). The influence of bioactive hydroxyapatite shape and size on the mechanical and biodegradation behaviour of magnesium-based composite. Ceram. Int..

[3] Madeira S., Barbosa A., Silva F.S., Carvalho O. (2020). Micro-grooved surface laser texturing of zirconia: surface characterization and artificial soft tissue adhesion evaluation. Ceram. Int..

[4] Heimann Robert B. (2021). Magnesium alloys for biomedical application: advanced corrosion control through surface coating. Surf. Coating. Technol..

[5] Moura Caroline Gomes, Faria D., Carvalho O., Santiago Floriani Pereira Rafael, Cerqueira M.F., Nascimento R.M., Samuel Silva Filipe (2020). Laser printing of silver-based micro-wires in ZrO2 substrate for smart implant applications. Opt Laser. Technol..

[6] Ji Min, Xu Jinyang, Chen Ming, El Mansori Mohamed (2020). Enhanced hydrophilicity and tribological behavior of dental zirconia ceramics based on picosecond laser surface texturing. Ceram. Int..

[7] Francis A.A., Abdel-Gawad S.A., Shoeib M.A. (2021). Toward CNT-reinforced chitosan-based ceramic composite coatings on biodegradable magnesium for surgical implants. J. Coating Technol. Res..

[8] Mao Bo, Siddaiah Arpith, Liao Yiliang, Menezes Pradeep L. (2020). Laser surface texturing and related techniques for enhancing tribological performance of engineering materials: a review. J. Manuf. Process..

[9] Mesquita-Guimarães J., Detsch R., Souza A.C., Henriques B., Silva F.S., Boccaccini A.R., Carvalho O. (2020). Cell adhesion evaluation of laser-sintered HAp and 45S5 bioactive glass coatings on micro-textured zirconia surfaces using MC3T3-E1 osteoblast-like cells. Mater. Sci. Eng. C.

[10] Zhang Zhao-Qi, Wang Li, Zeng Mei-Qi, Zeng Rong-Chang, Bobby Kannan M., Lin Cun-Guo, Zheng Yu-Feng (2020). Biodegradation behavior of micro-arc oxidation coating on magnesium alloy-from a protein perspective. Bioact. Mater..

[11] Bijukumar Divya Rani, Salunkhe Shruti, Zheng Guoxing, Barba Mark, Hall Deborah J., Pourzal Robin, Mathew Mathew T. (2020). Wear particles induce a new macrophage phenotype with the potential to accelerate material corrosion within total hip replacement interfaces. Acta Biomater..

[12] Jakubowska Ewelina, Gierszewska Magdalena, Nowaczyk Jacek, Olewnik-Kruszkowska Ewa (2020). Physicochemical and storage properties of chitosan-based films plasticized with deep eutectic solvent. Food Hydrocolloids.

[13] Rahman Mostafizur, Dutta Naba K., Choudhury Namita Roy (2020). Magnesium alloys with tunable interfaces as bone implant materials. Front. Bioeng. Biotechnol..

[14] Ali Murad, Mohamed Elsherif, Ahmed E., Salih Anwar, Ul-Hamid, Hussein M.A., Park Seongjun, Yetisen Ali K., Butt Haider (2020). Surface modification and cytotoxicity of Mg-based bio-alloys: an overview of recent advances. J. Alloys Compd..

[15] Cui Lan-Yue, Wei Guang-Bin, Han Zhuang-Zhuang, Zeng Rong-Chang, Wang Lei, Zou Yu-Hong, Li Shuo-Qi, Xu Dao-Kui, Guan Shao-Kang (2019). In vitro corrosion resistance and antibacterial performance of novel tin dioxide-doped calcium phosphate coating on degradable Mg-1Li-1Ca alloy. Journal of materials science & technology.

[16] Javed Rabia, Rais Farwa, Fatima Humaira, Ihsan ul Haq, Kaleem Muhammad, Sohaila Naz Syeda, Ao Qiang (2020). Chitosan encapsulated ZnO nanocomposites: fabrication, characterization, and functionalization of bio-dental approaches. Mater. Sci. Eng. C.

[17] Parvizifard M., Karbasi S. (2020). Physical, mechanical and biological performance of PHB-Chitosan/MWCNTs nanocomposite coating deposited on bioglass based scaffold: potential application in bone tissue engineering. Int. J. Biol. Macromol..

[18] Fu Jiayin, Su Yingchao, Qin Yi-Xian, Zheng Yufeng, Wang Yadong, Zhu Donghui (2020). Evolution of metallic cardiovascular stent materials: a comparative study among stainless steel, magnesium and zinc. Biomaterials.

[19] Kania Aneta, Pilarczyk Wirginia, Szindler Magdalena M. (2020). Structure and corrosion behavior of TiO2 thin films deposited onto Mg-based alloy using magnetron sputtering and sol-gel. Thin Solid Films.

[20] Wang Xiaoting, Guo Weiming, Li Lvyuan, Fei Yu, Li Jiayi, Liu Lu, Fang Bing, Xia Lunguo (2021). Photothermally triggered biomimetic drug delivery of Teriparatide via reduced graphene oxide loaded chitosan hydrogel for osteoporotic bone regeneration. Chem. Eng. J..

[21] Masud Rifat Ara, Islam Md Sazedul, Haque Papia, Khan M. Nazrul I., Shahruzzaman Md, Khan Mala, Takafuji Makoto, Mizanur Rahman Mohammed (2020). Preparation of novel chitosan/poly lycol)/ZnO bionanocomposite for wound healing application: effect of gentamicin loading. Materialia.

[22] Roshan Rahimi, Narges Hossein Hassannejad, Nouri Ashkan (2021). Corrosion and mechanical behaviour of biodegradable PLA-cellulose nanocomposite coating on AZ31 magnesium alloy. Surf. Eng..

[23] Xu Haitao, Hu Tu, Wang Manle, Zheng Yuxin, Qin Hui, Cao Huiliang, An Zhiquan (2020). Degradability and biocompatibility of magnesium-MAO: the consistency and contradiction between in-vitro and in-vivo outcomes. Arab. J. Chem..

[24] Rogowska-Tylman Julia, Locs Janis, Salma Ilze, Woźniak Bartosz, Pilmane Mara, Zalite Vita, Wojnarowicz Jacek (2019). In vivo and in vitro study of a novel nanohydroxyapatite sonocoated scaffolds for enhanced bone regeneration. Mater. Sci. Eng. C.

[25] Nowroozi Nona, Faraji Soraya, Nouralishahi Amideddin, Shahrousvand Mohsen (2021). Biological and structural properties of graphene oxide/curcumin nanocomposite incorporated chitosan as a scaffold for wound healing application. Life Sci..

[26] Rogowska-Tylman Julia, Locs Janis, Salma Ilze, Woźniak Bartosz, Pilmane Mara, Zalite Vita, Wojnarowicz Jacek (2019). In vivo and in vitro study of a novel nanohydroxyapatite sonocoated scaffolds for enhanced bone regeneration. Mater. Sci. Eng. C.

[27] Thirumalvalavan S., Senthilkumar N. (2020). Optimising the wear performance of HVOF thermal spray coated Ti-6Al-4V alloy by grey relational approach. Int. J. Rapid Manuf..

[28] Sundaraselvan S., Senthilkumar N., Tamizharasan T., Naveen Sait A. (2020). Surface modification of AZ61 magnesium alloy with nano TiO2/Al2O3 using laser cladding technique. Mater. Today: Proc..

[29] Bocchetta Patrizia, Chen Liang-Yu, Dias Corpa Tardelli Juliana, Andréa Cândido dos Reis, Almeraya-Calderón Facundo, Leo Paola (2021). Passive layers and corrosion resistance of biomedical Ti-6Al-4V and β-Ti alloys. Coatings.

[30] Gajalakshmi K., Senthilkumar N., Mohan B., Anbuchezhiyan G. (2020). An investigation on microstructure and mechanical behaviour of copper-nickel coated carbon fibre reinforced aluminium composites. Mater. Res. Express.

[31] Bibi Azeem, Akhtar Tasleem, Akhtar Kalsoom, Farooq Muhammad, Imran Shahzad Muhammad (2020). Alginate-chitosan/MWCNTs nanocomposite: a novel approach for sustained release of Ibuprofen. J. Polym. Res..

[32] Baktash M. Saviz, Ali Zarrabi, Avazverdi Ehsan, Nuno Miguel, Reis (2021). Development and optimization of a new hybrid chitosan-grafted graphene oxide/magnetic nanoparticle system for theranostic applications. J. Mol. Liq..

[33] Quazi Moinuddin Mohammed, Ishak Mahadzir, Fazal M.A., Arslan A., Rubaiee Saeed, Halil Aiman Mohd, Abdullah Qaban (2021). A comprehensive assessment of laser welding of biomedical devices and implant materials: recent research, development and applications. Crit. Rev. Solid State Mater. Sci..

[34] Chen Tao, Deng Zixin, Liu Defu, Zhu Xiangcheng, Xiong Yi (2021). Bioinert TiC ceramic coating prepared by laser cladding: microstructures, wear resistance, and cytocompatibility of the coating. Surf. Coating. Technol..

[35] Mukherjee Sumanta, Dhara Santanu, Saha Partha (2018). Laser surface remelting of Ti and its alloys for improving surface biocompatibility of orthopaedic implants. Mater. Technol..

[36] Baino Francesco, Angeles Montealegre Maria, Orlygsson Gissur, Novajra Giorgia, Vitale-Brovarone Chiara (2017). Bioactive glass coatings fabricated by laser cladding on ceramic acetabular cups: a proof-of-concept study. J. Mater. Sci..

[37] Chen Tao, Liu Defu, Wu Fan, Wang Haojun (2017). Effect of CeO2 on microstructure and wear resistance of TiC bioinert coatings on Ti6Al4V alloy by laser cladding. Materials.

[38] Lian G., Xiao S., Zhang Y. (2021). Multi-objective optimization of coating properties and cladding efficiency in 316L/WC composite laser cladding based on grey relational analysis. Int. J. Adv. Manuf. Technol..

[39] Lian G., Zhao C., Zhang Y., Feng M., Jiang J. (2020). Investigation into micro-hardness and wear resistance of 316L/SiC composite coating in laser cladding. Appl. Sci..

[40] Lian G., Liu Z., Zhang Y. (2022). Grey relational analysis–based composite coating property optimization fabricated by laser cladding. Int. J. Adv. Manuf. Technol..

[41] Lian G., Zhang H., Zhang Y., Tanaka M.L., Chen C., Jiang J. (2019). Optimizing processing parameters for multi-track laser cladding utilizing multi-response grey relational analysis. Coatings.

[42] Soni Raj, Pande Sarang (2022). Laser cladded Ti-alloys in biomedical applications: a review. Trends Biomater. Artif. Organs.

[43] Ibrahim Mahmoud Z., Ahmed A.D., Sarhan, Yusuf Farazila, Hamdi M. (2017). Biomedical materials and techniques to improve the tribological, mechanical and biomedical properties of orthopedic implants–A review article. J. Alloys Compd..

[44] Mantripragada Venkata P., Lecka‐Czernik Beata, Ebraheim Nabil A., Jayasuriya Ambalangodage C. (2013). An overview of recent advances in designing orthopedic and craniofacial implants. J. Biomed. Mater. Res..

[45] Bartel D.L., Bicknell V.L., Wright T.M. (1986). Effect of conformity, thickness, and material on stresses in ultra-high molecular weight components for total joint replacement. J Bone Joint Surg Am.

[46] Beillas P. (2004). A new method to investigate in vivo knee behavior using a finite element model of the lower limb. J. Biomech..

[47] Godest A.C. (2002). Simulation of a knee joint replacement during a gait cycle using explicit finite element analysis. J. Biomech..

[48] Moletsane Gloria, du Preez Willie, Nkhwa Shathani, Beer Deon (2023). Characterisation of bone-regenerating scaffolds produced through lithography-based ceramic manufacturing. S. Afr. J. Ind. Eng..

[49] Silva R., Santos M.D.d., Madureira R., Soares R., Neto R., Vieira Â.A., Gonçalves P.A.R., Leite P.M.S.M., Vieira L., Viana F. (2023). Scratch andWear behaviour of Co-Cr-Mo alloy in ringer's lactate solution. Materials.

